The article "Effect of the chemokine receptor CXCR7 on proliferation of carcinoma cells in vitro and in vivo" was retracted in 2011. Reason: concerns about the authorship.

# Effect of the chemokine receptor CXCR7 on proliferation of carcinoma cells *in vitro* and *in vivo*

**DOI:** 10.1038/sj.bjc.6604727

**Published:** 2008-10-14

**Authors:** J Meijer, J Ogink, E Roos

**Affiliations:** 1 Division of Cell Biology, The Netherlands Cancer Institute, 121 Plesmanlaan, 1066CX Amsterdam, The Netherlands

**Keywords:** tumour growth, chemokines, carcinoma, migration

## Abstract

The chemokine CXCL12/SDF-1 and its receptor CXCR4 have been implicated in invasion, survival and proliferation of carcinoma cells. Recently, CXCR7 was identified as a second receptor for CXCL12. We observed that CXCL12 promoted proliferation of CT26 colon and KEP1 mammary carcinoma cells, and this was blocked when CXCR7 was downregulated by ‘intrakines’ or RNAi, but not by CXCR4 inhibitors. The K1R mutant of CXCL12, which acts as a CXCR4 antagonist, also promoted proliferation through CXCR7 and is therefore a selective CXCR7 agonist. The effect of CXCR7 was not due to reduced apoptosis, and CXCR7 mediated chemotaxis of the carcinoma cells towards CXCL12. These results differ from those in a previous report on other carcinoma cells. We conclude that CXCL12 can be a potent growth factor for carcinoma cells by acting on CXCR7. Nevertheless, we observed no effect of complete and stable CXCR7 suppression on the growth of s.c. tumours or lung metastases of KEP1 and CT26 cells. A CXCR7 inhibitor has been reported to reduce growth of other tumours. Our results indicate that this inhibitor may not be applicable to therapy of all carcinomas.

CXCR4, the receptor of the chemokine CXCL12/SDF-1, is expressed in many tumours of multiple types including mammary (Muller *et al*, 2001), colon (Zeelenberg *et al*, 2003) and pancreatic (Saur *et al*, 2005) carcinoma, melanoma (Scala *et al*, 2005) and brain tumours (Rubin *et al*, 2003). Expression often correlates with the degree of malignancy and metastasis formation (Kaifi *et al*, 2005; Katayama *et al*, 2005; Kim *et al*, 2005; Scala *et al*, 2005; Schimanski *et al*, 2005). Indeed, CXCR4 was demonstrated to be required for experimental metastasis of mammary (Muller *et al*, 2001) and colon (Zeelenberg *et al*, 2003) carcinomas in the lungs and liver. In addition, CXCR4 was among a set of proteins that, in various combinations, promoted bone metastasis of mammary carcinoma cells (Kang *et al*, 2003). Furthermore, CXCR4 is induced by hypoxia and was proposed to be responsible for enhanced malignancy of tumour cells in hypoxic areas (Schioppa *et al*, 2003; Staller *et al*, 2003). This enhanced malignancy was generally attributed to a role of CXCR4 in invasion, as the ligand CXCL12 is present in many tissues and thought to promote migration into those tissues (Muller *et al*, 2001). We and others have shown, however, that chemokine receptors can also promote survival and proliferation of tumour cells (Barbero *et al*, 2003; Rubin *et al*, 2003; Zeelenberg *et al*, 2003; Katayama *et al*, 2005; Sutton *et al*, 2007; Yang *et al*, 2007). For CT26 colon carcinoma cells, we provided evidence that CXCR4 is required for the formation of liver and lung metastases, not because of enhanced invasion but rather due to an essential role in the outgrowth of the metastases (Zeelenberg *et al*, 2003).

To demonstrate this involvement of CXCR4 in the CT26 cells, we had expressed an ‘intrakine’ (Chen *et al*, 1997) that is the ligand CXCL12 extended with a C-terminal KDEL sequence. The intrakine binds to the KDEL receptor that retains resident proteins in the endoplasmic reticulum (ER). The intrakine is therefore retained in the ER, where it binds to newly synthesised CXCR4, which is also trapped. Thus, we generated cells without cell surface CXCR4 (Zeelenberg *et al*, 2001, 2003) that did not grow out in the lungs and liver. This intrakine approach was based on the generally held assumption that CXCR4 was the only receptor for CXCL12. Recently, however, the RDC1 protein was shown to be a second CXCL12 receptor and was renamed CXCR7 (Balabanian *et al*, 2005; Burns *et al*, 2006). It was described to be present on the surface of many tumour cell types and on activated endothelial cells. CXCR7 promoted the survival of tumour cells in minimal medium by preventing apoptosis and did not mediate chemotaxis towards CXCL12. Importantly, a CXCR7 inhibitor greatly reduced the growth of tumours generated from three different tumour cell lines (Burns *et al*, 2006).

The CXCL12-KDEL intrakine should bind CXCR7 and, similar to CXCR4, also trap CXCR7 in the ER. The results we obtained with the CT26 colon carcinoma cells might thus involve CXCR7 rather than, or in addition to, CXCR4. We therefore investigated this possible role of CXCR7 in the CT26 cells as well as in Panc02 pancreatic carcinoma and in KEP1 (knockout/E-cadherin/P53) mouse mammary carcinoma cells. The KEP tumours arose in p53 knockout mice in which the E-cadherin gene was disrupted in the skin and mammary glands. They are quite similar to human invasive lobular carcinomas with high metastatic capacity, and this behaviour is replicated by isolated KEP cells (Derksen *et al*, 2006). We found that CXCR4 is in fact the receptor required for metastasis. The cells do express CXCR7, however, and we observed CXCR7-mediated effects of CXCL12 that we describe here. We found that CXCL12 strongly enhanced proliferation, mediated by CXCR7, and on some cells, also by CXCR4. This chemokine is therefore a growth factor for carcinomas. Despite the strong *in vitro* effects, however, we observed no difference in growth rate *in vivo* of cells in which CXCR7 was completely and stably suppressed, at least not in s.c. tumours and lung metastases. This contrasts with the previously described effects of a CXCR7 inhibitor on other tumour cells, including a carcinoma (Burns *et al*, 2006). These observations are relevant for the consideration to use this receptor as a target for cancer therapy.

## Materials and methods

### Cell culture

The source of CT26 and Panc02 cells was described before (Meijer *et al*, 2006). KEP1 cells were kindly provided by Dr J Jonkers of the Netherlands Cancer Institute. All cells were cultured in DMEM with 10% FCS or in Keratinocyte medium with 1% FCS, both with 100 IU ml^−1^ of penicillin and 100 mg ml^−1^ of streptomycin. The Phoenix virus-packaging cell line (http://www.stanford.edu/group/nolan) was cultured in DMEM with 10% FCS and 0.584 g l^−1^ L-glutamine, the T-cell hybridoma TAM2D2 as described (Zeelenberg *et al*, 2001). Media, FCS and supplements were from Life Technologies Ltd, Paisley, UK.

### Generation and transduction of DNA constructs

The generation of the CXCL12-KDEL construct was described previously (Zeelenberg *et al*, 2001). CXCL12 cDNA was generated by PCR from this construct and the mutant K1R-CXCL12 from the K1R-CXCL12-KDEL construct (Zeelenberg *et al*, 2001). Both were cloned into the pLZRS-IRES-hygroEGFP vector (Zeelenberg *et al*, 2001). CXCL11-KDEL and CXCL10-KDEL were generated using a one-step RT–PCR kit (Qiagen, Valencia, CA, USA) on RNA isolated from mouse spleen, and inserted into the same vector. All constructs were checked by sequencing. Vectors were transfected into the virus-packaging Phoenix cells and the supernatant used to infect tumour cells. Transduced cells were selected with 0.05 (CT26) or 0.1 mg ml^−1^ (Panc02 and KEP1) hygromycin (Calbiochem-Novabiochem Corp., La Jolla, CA, USA) and cells with high GFP levels were isolated by FACS sorting. Control cells were transduced with the empty vector and sorted similarly. Luciferase was introduced as described (Meijer *et al*, 2006). The RNAi sequences GTGTTTCAATTCCAGCATA (CXCR4), CCCACTGTCTACTCAGGAA (CXCR7 RNAi.1: effective) and GAAATCATGTCCTTATCTT (CXCR7 RNAi.3: ineffective) were incorporated into the microRNA-30 sequence (Silva *et al*, 2005) and cloned into the LMP (MSCV/LTRmiR30-PIG) vector (Open Biosystems, Huntsville, AL, USA) that also contains the GFP cDNA under the control of the PGK promoter. For details see the literature provided by the supplier: http://www.openbiosystems.com/RNAi/RetroviralCloningVectors. The chosen sequences were derived from the RNAi Codex (http://codex.cshl.edu/scripts/newmain.pl). For transduction, we used Phoenix cells as above. Puromycin (1.75 *μ*g ml^−1^; Sigma-Aldrich, St Louis, MO, USA) was used for selection and cells with high GFP levels were FACS sorted.

### Generation of CXCR7 antiserum

The peptide DYAEPGNYSDINWP (mouse CXCR7, 7–21) was synthesised by the in-house facility and coupled to keyhole limpet haemocyanin. A polyclonal antiserum was generated in rabbits by standard procedures.

### Flow cytometry

Cultures were trypsinised and 10^6^ cells were incubated for 60 min with CXCR4 mAb 12G5 (R&D systems, Minneapolis, MN, USA) or with the CXCR7 antiserum and next with PE-conjugated antibodies against mouse or rabbit IgG, respectively, and analysed using a Becton Dickinson FACSCan using CellQuest software. Cells from tumours were isolated and treated as described (Meijer *et al*, 2006) and gated to exclude dead and GFP-negative cells so that only tumour cells that are GFP positive were analysed.

### Proliferation assay

CT26 cells (5 × 10^3^ or 10^4^ per well) or Panc02 or KEP1 cells (5 × 10^4^ per well) were seeded in several 96-well plates in DMEM with 10% FCS or Keratinocyte medium with 1% FCS. Luciferase activity was measured every 24 h after the addition of 10 *μ*l of 15 mg ml^−1^ D-luciferin, using a Xenogen IVIS imaging system (see below: *in vivo* bioluminescence). Each time, only one plate was measured and a different plate was assessed for each of the time points, so that each plate was measured only once. The data were normalised to 1 at day 0. As this assay did not involve any washing steps, it was quite reproducible, with standard deviations of triplicates of ∼0.02%. To some wells, 100 ng ml^−1^ CXCL12 (PeproTech Inc., Rocky Hill, NJ, USA) was added or supernatants of CT26 cells transfected with either CXCL12 or K1R-CXCL12 that had been grown in either 10 or 1% FCS. Supernatants of similarly cultured CT26 cells were used as controls. In some experiments, 125 ng ml^−1^ AMD3100 (Sigma, St Louis, MO, USA) or 1 ng ml^−1^ TC14012 was added. The TC14012 was synthesised by the in-house peptide facility.

### Apoptosis assay

Adherent cells were trypsinised and both the detached cells and those floating in the medium were collected, fixed with 70% ethanol, stained with propidium iodide and analysed by FACS, without gating. Cells in the G1 (*n*) and G2/M (2*n*) phases of the cell cycle could be distinguished. Apoptotic cells have a DNA content lower than *n*. As a positive control, apoptosis was induced by UV irradiation (50 J m^−2^, 16 h before the assay).

### Chemotaxis

For the carcinoma cells, chemotaxis was assayed as described (Meijer *et al*, 2006) with 100 ng ml^−1^ of CXCL12 in the lower well. Chemotaxis of T-cell hybridoma cells was measured as described (Zeelenberg *et al*, 2001).

### Tumour formation *in vivo*

All procedures involving animals were approved by the Animal Welfare Committee. For CT26 cells, we used syngeneic Balb/c mice and for KEP1 cells, nude mice, both 6–8 weeks old. Cells (10^3^) were dispersed in 0.5 ml Matrigel (Becton Dickinson, Franklin Lakes, NJ, USA) at 0°C and injected s.c. into mice anaesthetised with 3% 1-chloro-2,2,2-triflouroethyl-diflouromethyl-ether (isoflurane). Alternatively, we injected 0.2 ml PBS containing 10^5^ cells into a tail vein or 0.1 ml containing 10^6^ cells subcutaneously.

### *In vivo* bioluminescence imaging

D-Luciferin (Xenogen, Alameda, CA, USA) was dissolved at 15 mg ml^−1^ in sterile PBS and stored at −20°C. Animals were anaesthetised with 3% isoflurane. Luciferin solution was injected i.p. (0.01 ml per g body weight). Light emission was measured 5 min later, using a cooled CCD camera (IVIS; Xenogen), coupled to Living Image acquisition and analysis software over an integration time of 2 min. Signal intensity was quantified as the total counts measured over the region of interest.

## Results

### CXCL12 promotes proliferation of CT26 carcinoma cells, but not through CXCR4

We have previously shown that CT26 colon carcinoma cells require CXCR4 for outgrowth of metastases (Zeelenberg *et al*, 2003). The cells have no surface CXCR4 *in vitro* (see Figure 1C) but acquire it *in vivo*. The cells do not express the CXCR4 ligand CXCL12, as determined by RT–PCR (data not shown). We reasoned that if these cells would produce this ligand, *in vivo* growth of metastases might be further promoted, and therefore we transfected the CXCL12 cDNA. Much to our surprise, the resulting CXCL12-producing cells proliferated faster than control CT26 cells *in vitro*, despite the absence of CXCR4. In addition, we transfected the K1R mutant of CXCL12, which is a potent inhibitor of CXCR4 (Crump *et al*, 1997). Remarkably, the mutant also increased proliferation. This indicated that the increase in proliferation was mediated by an, at the time, unknown second CXCL12 receptor.

To demonstrate that the effect was due to the expressed proteins, the supernatants were added to wild-type CT26 cells. Proliferation was increased by both supernatants to a similar extent as recombinant CXCL12 (Figure 1A). This was not only seen in minimal medium (1% FCS) but also in optimal medium (10% FCS) in which proliferation was already quite fast. In either of these circumstances, the percentage of apoptotic cells was very low, as assessed by FACS analysis of propidium iodide-stained cells (Figure 1C). The percentage varied between 1 and 4%, as compared with ∼50% in UV-irradiated cells that were used as positive controls, and was not lower in CXCL12-treated cells, showing that the effect could not be due to the suppression of apoptosis.

To confirm that the K1R mutant is a CXCR4 inhibitor, we studied chemotaxis of TAM2D2 T-cell hybridoma cells (Zeelenberg *et al*, 2001) towards CXCL12. As shown in Figure 1B, this is blocked by the CXCR4 inhibitors AMD3100 (Donzella *et al*, 1998) and TC14012 (Tamamura *et al*, 2001), and therefore mediated by CXCR4. K1R-CXCL12 did not induce chemotaxis and it inhibited chemotaxis towards intact CXCL12, confirming that it is a CXCR4 antagonist. The two CXCR4 inhibitors did not influence the CXCL12-induced enhancement of proliferation of CT26 cells at concentrations at which they completely inhibited chemotaxis mediated by CXCR4 (Figure 1B).

The CXCL12 concentration in the supernatant was ∼100 ng ml^−1^, based on a comparison of dose–response curves with recombinant CXCL12 (data not shown). The mutant was expressed at similar levels, as deduced from co-expressed GFP, and its concentration in the supernatant is likely roughly comparable, as deduced from ∼35% inhibition of chemotaxis towards 100 ng ml^−1^ CXCL12 (Figure 1B). For proliferation, concentrations were saturating, as the effect was the same at 50% dilution. For both, the effect was reduced by ∼60% at 10% dilution (data not shown), indicating that the affinity for CXCR7 was comparable.

### Effect of CXCL12 on proliferation of CT26 cells is mediated by CXCR7

While this work was in progress, the identification of a second CXCL12 receptor was reported: the orphan receptor RDC1/CMKOR1, which was renamed CXCR7 (Balabanian *et al*, 2005; Burns *et al*, 2006). We established by RT–PCR that CT26 and KEP1 cells expressed CXCR7 (data not shown). Next, we generated a polyclonal antiserum against a peptide that is the mouse homologue of the epitope of an anti-human CXCR7 mAb (Balabanian *et al*, 2005). Using this antiserum, we detected CXCR7 on the surface by FACS analysis. As shown in Figure 1C, CT26 cells that were devoid of CXCR4 did express CXCR7 *in vitro*.

Next, we tested CXCL12 on KEP1 mammary carcinoma cells (Derksen *et al*, 2006). The KEP1 cells did express not only CXCR4 *in vitro*, but also CXCR7 (Figure 2A). They grow slower than CT26 cells, but again we observed enhanced proliferation although the effect was somewhat less pronounced than in CT26 cells (Figure 2B), and the extent of stimulation was again similar in 1 and 10% FCS. The data shown in Figure 2B were from cells in 1% FCS. The K1R mutant had a similar effect (Figure 2B), indicating that CXCR4 was not involved. The concentration of the ligands was saturating, as a 50% reduction led to identical results. CXCL12 similarly enhanced the proliferation of human carcinoma cell lines, including CAPAN1 pancreatic carcinoma and MDA-MB-231 mammary carcinoma (data not shown). The MDA-MB-231 variant we used did not express CXCR4 *in vitro*, again showing that CXCR4 was not involved.

RNAi would have been the most straightforward approach to discriminate between functions of CXCR4 and CXCR7. As this was initially not successful, and also to obtain independent evidence, we again used the intrakine approach (see Introduction). As CXCR7 also binds CXCL11, whereas CXCR4 does not (Burns *et al*, 2006), a CXCL11-KDEL intrakine should trap CXCR7 in the ER selectively. However, CXCL11 also binds the CXCR3 chemokine receptor that may be expressed by carcinoma cells (Goldberg-Bittman *et al*, 2004). We therefore used a CXCL10-KDEL intrakine as control, because CXCL10 also binds CXCR3 but not CXCR7 (Burns *et al*, 2006). We could not express either of these intrakines in CT26 cells even though we did successfully transfect several other intrakines: CXCL12-KDEL (Zeelenberg *et al*, 2003), CXCL13-KDEL (Meijer *et al*, 2006) and recently, also CXCL16-KDEL (Meijer *et al*, 2008), in these cells. This suggested that CXCR3 is required for their survival and/or growth. However, we did express the two intrakines in KEP1 cells and both at similar levels, as determined by FACS analysis of GFP that was co-expressed from the bicistronic vector. CXCL11-KDEL completely blocked transport to the cell surface of CXCR7, but not CXCR4, resulting in cells without cell surface CXCR7 (Figure 2A). CXCL10-KDEL had no such effect (Figure 2A). The CXCR7-deficient cells did not respond at all to intact or mutant CXCL12 (Figure 2B), providing strong evidence that CXCR7 was the involved receptor. CXCL12-KDEL downregulated both CXCR4 and CXCR7 (Figure 2A), and because of the latter effect also blocked the (K1R)-CXCL12-induced proliferation (Figure 2B).

Later, we did achieve knockdown of CXCR7 using an shRNAmir vector that encodes a natural microRNA containing the RNAi sequence (Silva *et al*, 2005). Sorting for high levels of co-expressed GFP yielded KEP1-RNAi.1 cells in which CXCR7 was completely suppressed (Figure 2A). As a control, we used another CXCR7 sequence (RNAi.3) that was completely ineffective (Figure 2A), as well as a CXCR4 RNAi that completely suppressed CXCR4 but not CXCR7 (Figure 2A), all expressed at similar levels as based on GFP fluorescence (not shown). Again, the CXCR7-deficient cells did not respond at all to CXCL12, whereas the control cells did (Figure 2B), demonstrating that CXCR7 is the involved receptor. CXCR7 RNAi.1 had the same effect in CT26 cells (not shown).

### Both CXCR7 and CXCR4 enhance proliferation in Panc02 pancreatic carcinoma cells

We next tested Panc02 pancreatic carcinoma cells that express both CXCR4 and CXCR7 (Figure 3A). However, the CXCR7 levels were lower than on KEP1 cells, whereas the CXCR4 levels were comparable or higher (compare Figures 2A and 3A). Again, CXCL12 enhanced proliferation (Figure 3B and C). In these cells, this was mediated by both CXCR7 and CXCR4, as a complete knockdown of either (Figure 3A) caused a partial inhibition (Figure 3B and C), whereas the CXCL12-KDEL intrakine, which completely eliminated both from the surface (Figure 3A), reduced proliferation to control levels (Figure 3B). In line with this notion, K1R-CXCL12 had a smaller effect than intact CXCL12, and this was fully blocked by CXCR7 but not CXCR4 knockdown (Figure 3D), again showing that the K1R-CXCL12 mutant activates only CXCR7. We conclude that both receptors can trigger growth-promoting signals.

In all these experiments, proliferation was measured by bioluminescence. As this involves no washing steps, the data are quite reproducible with s.e.m. of ∼0.2%. The CXCL12-induced increases in cell number observed after 7 days were therefore always highly significant (*P*<0.0001). To demonstrate that bioluminescence reflects cell number, we trypsinised the cells from the wells after measuring bioluminescence and counted the cells. An example is given in Figure 3C. The results were similar and the *P*-values of the differences were <0.0001.

### CXCR7 mediates chemotaxis towards CXCL12

CXCR7 was reported to differ from CXCR4 in that it did not induce chemotaxis towards CXCL12 (Burns *et al*, 2006). We tested this using the CXCR4-negative CT26 cells and found that CXCL12 potently induced chemotaxis, which was not inhibited by the CXCR4 inhibitors AMD3100 and TC14012 (Figure 4A). Chemotaxis was maximal at 100 ng ml^−1^ and half-maximal at 40 ng ml^−1^ (not shown). The K1R CXCR4 mutant was equally effective, showing again that it is a CXCR7-specific agonist. Migration was inhibited by 60% in cells in which Gi protein signalling was fully blocked by pertussis toxin, showing that it is mediated by both Gi-dependent and Gi-independent mechanisms (not shown). Cells expressing CXCL12-KDEL or CXCR7-RNA.1, in which CXCR7 was suppressed, did not migrate towards CXCL12 (Figure 4B). CXCR4 RNAi had no effect, as expected for cells that do not express CXCR4 *in vitro*. This chemotaxis was comparable to the extent to that induced by CXCL11 (not shown). This was reduced by ∼50% by CXCR7 RNAi, the remainder likely due to CXCR3, the presence of which was not further studied. We conclude that CXCR7 signals are clearly able to trigger migration but that this apparently depends on the cell type.

### No effect of CXCR7 on tumour growth *in vivo*

To test the effects on growth *in vivo*, we subcutaneously injected cells in Matrigel. On account of the instant solidification at 37°C, cells remained dispersed and initially grew as separate single tumours. All cells expressed luciferase and growth was monitored by measuring bioluminescence after the injection of luciferin. As shown in Figure 5A, KEP1 control cells (expressing GFP from an empty vector) and other CXCR7-positive KEP1 controls (the ineffective CXCR7 RNAi.3 and CXCL10-KDEL) grew at the same rate as the CXCR7-deficient cells (CXCR7 RNAi.1 and CXCL11-KDEL). The Td for controls was 54.3 h (s.e.m., 0.7) and for the CXCR7-deficient cells 53.1 h (s.e.m., 0.8). The difference was clearly not significant (*P*=0.27). In cells isolated from tumours 4 weeks after injection, CXCR7 was still completely suppressed (Figure 5B). (Please note that the FACS profiles differ from those *in vitro* (see Figure 2), quite likely due to the collagenase treatment. The relevant comparison is with control cells of which the CXCL10-KDEL cells are shown).

This lack of effect might be due to the Matrigel that might contain factors that compensate for the lack of CXCR7 signalling. We therefore injected cells subcutaneously, without Matrigel, similarly as the Lewis lung carcinoma cells of which the growth was reported to be reduced by a CXCR7 inhibitor (Burns *et al*, 2006). Again, we saw no effect of CXCR7 deficiency (Figure 5C). The growth rate was remarkably similar to that in Matrigel: Td=54.0 h (s.e.m., 1.1) for controls and 54.0 h for the CXCR7-deficient cells (s.e.m., 1.4; *P*=0.48). Finally, we injected CT26 cells into a tail vein and found that lung metastases of CXCR7-deficient cells grew at the same rate as control cells (Figure 6A). The Td for controls was 73.2 h (s.e.m., 3.6) and for the CXCR7-deficient cells, it was 77.2 h (s.e.m., 1.2). The difference was not significant (*P*=0.34). We conclude that the presence of CXCR7 does not lead to enhanced proliferation *in vivo*, at least not in s.c. tumours and in lung metastases. The tumour cells were isolated from lung metastases after 24 days and analysed by FACS (Figure 6B). Thus, we confirmed our previous observation (Zeelenberg *et al*, 2003) that CT26 cells, which are devoid of CXCR4 *in vitro*, do express CXCR4 *in vivo*. Furthermore, we found that CXCR7 was still completely suppressed in the CXCR7-RNAi cells, so that the lack of effect on growth is not due to loss of the RNAi effect during the experiment.

## Discussion

CXCR7, the newly discovered second receptor of CXCL12, was reported to be expressed by several different tumour cell types and to mediate a CXCL12-induced increase of survival of mammary carcinoma cells in minimal medium. CXCR7 did not promote proliferation (Burns *et al*, 2006). We show here that these conclusions are not generally valid for carcinomas. In mouse CT26 colon, KEP1 mammary and Panc02 pancreatic carcinoma cells, CXCL12 increased proliferation and this was mediated by CXCR7, as we conclude based on the following observations. First, CT26 cells express CXCR7 but not CXCR4 *in vitro*. Second, the K1R mutant of CXCL12, which is a CXCR4 antagonist (Crump *et al*, 1997), also induced proliferation. Third, downregulation of CXCR7, by either the CXCL11-KDEL intrakine or RNAi, abolished the effects. CXCL10-KDEL (that should affect CXCR3, if present, similarly as CXCL11-KDEL) and an ineffective RNAi sequence served as controls that were expressed at similar levels but did not inhibit.

It is particularly noteworthy that the K1R mutant of CXCL12 triggers CXCR7. Lysine at position 1 in CXCL12 is not required for binding to CXCR4, but is essential for the triggering of CXCR4 signals (Crump *et al*, 1997). The K1R mutant binds CXCR4 but does not signal and therefore acts as a powerful antagonist. Indeed, it strongly inhibited the chemotaxis of T-cell hybridoma cells towards CXCL12. In contrast, it enhanced proliferation, by activation of CXCR7, to a similar extent as the intact chemokine. K1R-CXCL12 is therefore a selective agonist for CXCR7.

CXCR7 is not the only CXCL12 receptor that can trigger enhanced growth. CXCR4 can also mediate this effect, as demonstrated using specific inhibitors and antibodies (Barbero *et al*, 2003; Rubin *et al*, 2003; Katayama *et al*, 2005; Sutton *et al*, 2007; Yang *et al*, 2007). In fact, we show here that in Panc02 pancreatic carcinoma cells, CXCR4 contributes to the CXCL12-induced enhancement of proliferation. In KEP1 cells, the effect is mediated exclusively by CXCR7. This may be due to the relatively high CXCR7 levels (compare Figures 2A and 3A).

It was previously reported that the number of MDA-MB-435 human mammary carcinoma cells expanded in the presence of CXCL12, an effect mediated by CXCR7 (Burns *et al*, 2006). This occurred in minimal medium containing only 1% FCS, in which extensive apoptosis was observed in the absence of CXCL12. The increase in cell number was due to the prevention of apoptosis by the CXCR7 signals, and apparently not due to an enhanced proliferation. Our results with the CT26 and KEP1 cell lines were quite different. We observed only minimal apoptosis in 1% FCS. Moreover, an equally strong increase in proliferation occurred even in ‘optimal’ medium containing 10% FCS. Furthermore, it was reported that CXCR7 did not mediate chemotaxis of MCF-7 mammary carcinoma cells towards CXCL12 (Burns *et al*, 2006). This is, however, not generally true as the CXCR4-negative CT26 colon carcinoma cells did migrate towards CXCL12, mediated by CXCR7, as was in fact previously demonstrated for T lymphocytes (Balabanian *et al*, 2005). We conclude that CXCR7 is able to initiate powerful proliferation- and migration-inducing signals, but that the response apparently differs between cell types. Furthermore, we conclude that the chemokine CXCL12 can act as a powerful growth factor by signals transmitted by either or both CXCR4 and CXCR7. This adds to our previous observation that the chemokine CXCL13 can act as a growth factor for carcinoma cells that express its receptor CXCR5 (Meijer *et al*, 2006), suggesting that chemokines may be more generally involved in tumour growth.

Surprisingly, despite the strong *in vitro* effects, CXCR7 did not influence tumour growth *in vivo*, at least not in s.c. tumours and in lung metastases. Both the CXCL11-KDEL intrakine and RNAi caused complete and stable downregulation of CXCR7, but neither had any effect on growth rates in s.c. Matrigel plugs *in vivo*. This might be attributed to the absence of CXCL12 in these artificially induced tumours, which may lack the proper tumour environment. Supplying the ligand did not seem to have an effect either, however, as the CT26 cells in which CXCL12 or the selective CXCR7 agonist K1R-CXCL12 was expressed did not grow faster *in vivo* (data not shown), although we can not be sure that production of these chemokines was actually maintained *in vivo*. Importantly, we also found no evidence for CXCR7 involvement in s.c. tumours, established in a manner comparable with the Lewis lung carcinomas that were shown to be affected by a CXCR7 inhibitor (Burns *et al*, 2006). Finally, also growth of lung metastases was not influenced by the suppression of CXCR7.

Recently, *in vivo* effects of CXCR7 RNAi on other tumours were reported (Miao *et al*, 2007). Tumour growth was reduced to different extents. For instance, the final tumour weight of s.c. Lewis lung carcinomas was reduced by ∼50%, whereas the effect on 4T1 mammary carcinoma was larger. Our results clearly indicate that this is not generally applicable to carcinomas, at least not in s.c. tumours or lung metastases. This does not exclude an effect of CXCR7 in other circumstances. In fact, the expression of CXCR7 on many tumour cells and the ubiquitous presence of CXCL12 in tissues suggest that this should occur, perhaps in tissues that are particularly rich in CXCL12 or in particular stages of tumour development. It may also depend on whether, and to what extent, the tumour cells produce autocrine CXCL12. It should, however, not be expected that CXCR7 inhibitors would be applicable to therapy of all carcinomas.

## Figures and Tables

**Figure 1:** (**A**) Proliferation of CT26 colon carcinoma cells in supernatants of CT26 cells, either or not supplemented with 100 ng ml^−1^ recombinant CXCL12, or in supernatants of CT26 cells expressing CXCL12 or the K1R-CXL12 mutant. The supernatants contained either 1 or 10% FCS. Changes in cell numbers were measured by bioluminescence of these luciferase-expressing cells, after the addition of luciferin. Shown are the results of one of the two experiments with virtually identical results. The s.e.m. are extremely small (∼0.02%) and error bars are therefore not shown. For clarity, we used markers that are far larger than the error bars, and they were slightly displaced when overlapping to make them all visible. (**B**) Verification of effects on CXCR4 by CXCR4-mediated chemotaxis of TAM2D2 T-cell hybridoma cells in 2 h towards different concentrations (ng ml^−1^) of recombinant CXCL12, towards supernatants (sup) of control CT26 cells or of CXCL12- or K1R-CXCL12-expressing CT26 cells, or to 100 ng ml^−1^ CXCL12 added to the K1R-CXCL12-containing supernatant. AMD3100 (125 ng ml^−1^) and TC14012 (1 ng ml^−1^) inhibit completely at these concentrations, whereas they have no effect on CXCL12-induced proliferation. Shown are the results of one of the four experiments with similar results. (**C**) FACS analysis of CXCR4 and CXCR7 on CT26 cells grown *in vitro* and of PI-stained cells, either UV-irradiated or not 16 h before.

**Figure 2:** (**A**) Effects of intrakines or RNAi on CXCR4 and CXCR7 surface levels of KEP1 mammary carcinoma cells. Open histograms: negative controls (second antibody only for CXCR4 or preimmune serum and second antibody for CXCR7). Grey filled histograms: either CXCR4 mAb (upper row) or CXCR7 antiserum (lower row). (**B**) Effect of intrakines and RNAi on proliferation of KEP1 cells in 1% FCS-containing supernatants, as in Figure 1. Concentrations of both CXCL12 and mutant were saturating, as the effects were similar at 50% dilution (not shown). Results are from one of the two experiments with virtually identical results.

**Figure 3:** (**A**) Effects of intrakines or RNAi on CXCR4 and CXCR7 surface levels of Panc02 pancreatic carcinoma cells. Open histograms: negative control (preimmune serum and second antibody for CXCR7). Grey filled histograms: CXCR4 mAb; black filled histograms: CXCR7 antiserum. For clarity, only the negative control for the polyclonal antiserum is shown. Therefore, the fluorescence of CXCR4-suppressed cells seems lower than this control. In reality, they coincide with the proper control. (**B**) Proliferation of these cells in the presence or absence of 100 ng ml^−1^ CXCL12, as measured by bioluminescence. (**C**) The number of cells per well after 7 days in the same experiment as in panel B, manually counted after trypsinisation. (**D**) The effect of CXCL12-KDEL intrakine and CXCR4 or CXCR7 RNAi on the proliferation of Panc02 cells in supernatants of control or CXCL12- or K1R-CXCL12-expressing CT26 cells, as in Figure 1A. Results in panels B–D are of one of the three experiments with almost identical results.

**Figure 4:** Chemotaxis of CT26 colon carcinoma cells in 6 h towards 100 ng ml^−1^ CXCL12. (**A**) In the presence or absence of the CXCR4 inhibitor AMD3100 (125 ng ml^−1^) or TC14012 (1 ng ml^−1^). Data shown are of one experiment of two with similar results. (**B**) The effect of CXCL12-KDEL intrakine and CXCR4 or CXCR7 RNAi. Results are averages of two experiments. Error bars represent s.e.m.

**Figure 5:** Effect of CXCR7 suppression on growth of KEP1 mammary carcinoma cells *in vivo*. (**A**) In Matrigel plugs. CXCR7-positive controls: untransfected, CXCL10-KDEL and CXCR7-RNAi.3 (see Figure 2A), *n*=2 for each, total *n*=6. CXCR7-negative cells: CXCR7-RNAi.1, CXCL11-KDEL (see Figure 2A), *n*=2 for each, total *n*=4. Error bars represent s.e.m. (**B**) CXCR7 levels on cells isolated from plugs. Note that background is higher for these collagenase-treated cells than for untreated cultured cells (compare negative controls with Figure 2A). The profile of CXCR7-deficient cells coincides with the negative controls, showing that the effects of intrakine and RNAi are stable for at least 4 weeks *in vivo*. (**C**) The growth of s.c. injected cells (without Matrigel), as in panel A. CXCR7-deficient cells now also include cells expressing CXCL12-KDEL. Total of both control and deficient cells, *n*=6.

**Figure 6:** (**A**) Proliferation of lung metastases of CT26 colon carcinoma cells after tail vein injection of mice with control cells (*n*=5) or CXCR7-deficient cells (CXCR7 RNAi.1, *n*=5). Error bars represent s.e.m. (**B**) FACS analysis of CXCR4 and CXCR7 in CT26 cells isolated from lung metastases after 24 days. Although the cells are devoid of CXCR4 *in vitro*, they do express CXCR4 *in vivo*. The complete suppression of CXCR7 by RNAi is maintained throughout these 24 days.
